# Research on Competition and Cooperation Relationship of TV-Drama Production Company Based on Social Network

**DOI:** 10.1155/2022/9913269

**Published:** 2022-10-03

**Authors:** Zhongren Zhao, Peiyi Song, Yan Xu

**Affiliations:** ^1^School of Economics and Management, Communication University of China, Beijing 100024, China; ^2^ReachTop Education School, Beijing 100080, China

## Abstract

The social network is affecting the connection of TV-drama production companies, and traditional partnerships are changing. Many companies are moving from traditional connections to gridded social networks. The changing relational network makes the relationship between TV-drama production companies change from linear and static to network and dynamic, and from the original cooperation based on “Contract” to the node-type cooperation of “Switch.” Through empirical study, the paper found that the social network relationship in the TV series production industry has become an essential social capital because the construction of social networks will effectively promote the development of the industry under the new competition and make TV-drama industry production chain, creative resources, and value derived channel, resource boundary and cooperation mechanism, and market competition pattern change. Ultimately, it will reshape the subject cognition, path cognition, and power cognition in the relationship network.

## 1. Introduction

As top video websites such as IQiyi, YouKu, and Tencent Video increase the purchase and self-production of Internet Drama due to competition, some small production companies can participate in drama production, which activates the part of the long tail production market of the TV-drama industry. However, Chen considered that small companies cannot support the large investment compared with big companies in TV-drama production, and even they have a declining trend in the production chain [1]. The small company is changing from participants in enterprise cooperation to implementers or workers in a cooperative network, only participating in a certain kind of work in the project. As the production cost of TV-drama increases year by year, the market dislocation of production and sales brings great pressure to TV-drama production companies. Many TV dramas cannot be broadcast after shooting, resulting in losses for TV-drama production companies.

In 2021, The State Broadcasting and Television Administration of China announced the collection of Film and Television Production License in 2021–2023. Only 41 companies received the licenses in 2021, down 44% from 71 in 2019. It shows not only that the total number of TV-drama production companies is shrinking, but also that the TV-drama production market is extremely competitive. If some small companies want to participate in TV-drama production, they need to rely on or unite with large companies to share the benefit and development dividend of TV-drama industry. “Association” means relationship management. In Chinese society, the relationship has always been the main characteristic of Chinese people to get along with, not to mention the interest exchanges between enterprises. Fei describes Chinese society as a “Network” of relationships and human relationships society, which is centered on a certain subject and spread out according to the distance and strength of the relationship [2]. This also shows that the economic behavior of enterprises is bound to be influenced by social relations, and in today's complex Internet society, the influence is more profound. Therefore, research on enterprise behavior based on relationships and social network is of great value in Chinese society.

## 2. Literature Review

In the current era of reform and innovation, enterprises hope to find different organizations in the market to realize the integration of internal and external resources through cooperation and create content or products with greater value. Especially in the rapid change and innovation of TV-drama industry today, innovation cooperation is the only way to ensure the healthy development of TV-drama industry. Zhang argued that creative businesses do not only have sufficient capital, knowledge, and skills in traditional resources, but also need to be able to develop themselves as the main body, embedded in the industry, both inside and outside of different enterprises to establish a social relation network, to learn to rely on network nodes to help the company achieve its goals [3].

Regarding the cultural and creative industry as one part of the strategy of developing a strong culture, many scholars of communication, economics, and geography have begun to pay attention to the industrial network mode with “cultural projects” as the core of participation [4]. He et al. noted that network nodes and main body connections of the cultural and creative industry are mostly concentrated in the interior divided by cities, ignoring external connections that can accelerate the development of the cultural and creative industry [5]. Xin et al.'s study found that the film industry was divided into “Spokes” structure on the edge and core of the relational network, and they gave the analysis of the core node, such as the China film group, which is the core of the resource-exhausted state-owned enterprises that occupy the network, and Beijing as China's film industry agglomeration corresponding type of center city [6]. Wen et al. selected the 318 TV dramas on Television Station and the Internet as the research objects and analyzed the network structure in the space cooperation of the main producer. They found that, in the production chain of Internet Video, producing company location, core city nodes, and the connection degree among cities have gathered phenomenon. By these three indicators, the Beijing-Tianjin-Hebei region and the Yangtze River Delta region are the prominent areas [7].

Relational organization characteristics of TV-drama industry are obvious. The traditional mode of “enterprise cooperation” is challenged in the era of network economy, and TV-drama production companies outside the relationship network appear to be alone and lack competitiveness [8]. In particular, the characteristic of modular production in the TV-drama industry is remarkable. Johns believed that the relational network formed between TV-drama production companies based on the division of the industrial chain has become the main mode of TV-drama production [9]. This also coincides with the “social network market” theory of creative industry proposed by Janson Potts and John Hartley, which was originally proposed to explain the “user-led innovation” mode in the new media era [10]. With the development of the creative industry, they also believe that the relationship between actors, networks, and enterprises in the creative industry is a dynamic structure that allows them to help each other. Every writer or artist is an actor, every organization or company is a producer, and every connection is a network [11]. This theory breaks the traditional standard of distinguishing industry competitiveness through input and output, puts the social network in the core position of market development, and shows the relationship network model of the creative industry [12]. For any TV series, from the beginning of creativity to the final broadcast, all the links involved in the shooting, production, production, publicity, distribution, broadcasting, and other links need to be jointly completed by different participants in the network [13].

Many other scholars pay more attention to the TV-drama industry from different views as well, such as mode innovation and format change, but most of the discussions focus on the operation level, and the analysis of network relationship is insufficient. Social network theory just provides us with a tool to understand the relationship behind the TV-drama production company. The following four questions are discussed in this paper:

- How do social relationship networks behave in reality?
- Is there a network faction in the relationship between drama production companies?
- Does relying on core nodal companies to build network relationships mean the enhancement of competitiveness?
- Should future TV production companies build relationships to enhance their competitiveness?

## 3. Methodology

### 3.1. Social Network Analysis

Social network analysis (SNA) has become an important research method in sociology and behavioral sciences. SNA mainly focuses on the relationship between social agents (such as information exchange between groups) and relies on statistical methods and visual means to realize the image presentation of group relations [14]. When social networks were studied in the first stage of sociology, it was more about observing static systems, including the connections between network nodes and network individuals and their quantitative relationships. In recent years, social networks, combined with statistical physics, have begun to pay more attention to large networks, including the topology of networks and the dynamics of internal search commonalities that control their evolution [15].

Afterwards, the social network approach is increasingly used as a structured method to analyze informal relationships in formal organizations, including between people, teams, departments, and even organizations [16]. Social network analysis can help identify effective groups by transforming intangible relationships into tangible interactive structures [17]. Therefore, the method of social network has certain value in the evaluation of organization cooperation in film and television industry.

Recently, the social network method has been frequently used in various fields of research. A search on SCOPUS using the keyword “social network analysis” revealed over 2000 articles using SNA; for example, in supply chain studies [18], film industry studies [19], and health and medicine industry studies [20], social network methods are widely used.

In this study, we use social network analysis to expose the corporate partnerships behind the TV-drama industry, to find the key organizations in the TV-drama industry. The data used in this paper are all from real TV series projects, taking TV series coproduction as the target relationship research object, and exploring the production network structure of TV series industry through the interpretation of social network indicators.

### 3.2. Relationship and Information Sharing Model

In the age of information, the cooperation mode among supply chain enterprises in the TV-drama industry is developing rapidly, and the information sharing and timeliness of information among supply chain enterprises have been widely concerned and studied by scholars [21]. In traditional industries, such as manufacturing [22] and energy [23], their information sharing in the supply chain mainly solves the problem of technology adoption and technology absorption, but for cultural industries, the value of information itself and the way of information sharing are more important to the development of industrial project. In the TV-drama industry social network based on cooperation, timeliness and accuracy of information are the bases of getting added value for each company in the supply chain [24].

Lee et al. [25] proposed a two-layer value creation model of supply chain information sharing. They believed that, by sharing demand information, manufacturers could effectively reduce inventory level and inventory cost and reduce bullwhip effect. In order to highlight the effect of information sharing, the conclusion of Lee's mode is established on the basis that information sharing has no cost, and the quality of shared information is extremely high. On the basis of Lee's study, some subsequent researchers demonstrated the value of information sharing from different perspectives [26–29].

For TV-drama industry, information integration and information sharing between supply chain enterprises are important factors in TV-drama projects to achieve output value. The performance level of TV-drama project is affected by the information integration and information sharing [30]. Information sharing degree also directly affects the income of TV-drama supply chain participants. However, in the process of information collection and sharing, in addition to the necessary technical system support, the mutual trust between TV-drama social network members is the premise of cooperation. Especially in the context of social production in China, social network relationship is a potential element of Chinese culture that cannot be ignored, and this relationship can have an important impact on interpersonal trust and individual behavior decision-making [31]. Therefore, there is a significant correlation between social network relationships and supply chain performance in supply chain management.

With the help of the information asymmetry hypothesis in information economics [32], this paper constructs one model of relationship and information delivery (Figure 1) between the production subjects of the TV-drama industry supply chain, in which the timeliness and accuracy of information are fully considered.

In the model, the accuracy of information refers to the similarity between the shared information of the system and the actual information, that is, the degree to which it reflects the real situation. Information timeliness refers to the time delay of information occurrence when it is collected and transferred to use, and it is also the instantaneous acquisition ability of information.

## 4. Analysis and Finding

Starting from the connection between people, the relational network has almost become the main form of human social communication in the information age and provides a new way for enterprises to grasp the needs of the audience. As we all know, there is a relational network positioning based on users and business relationships on Facebook, which helps enterprises “establish relationships” with users through their home pages, applications, or activities. Enterprises can match or shield relationship types according to their goals, so that advertisements can be targeted accurately [33].

In the 1830s, Professors Joe and Scherer of Harvard University developed a framework model for industrial analysis, which described the relationship between market structure, firm behavior, and market performance [34]. Market structure is the structure of the relationship between market participants. This kind of “relationship” can be traced back to the “relationship” in the basic unit of social structure proposed by Georg Simmel, a German classical sociologist. He believed that a social relationship is a form of interaction between social subjects [35]. At present, it can be understood that enterprises, as actors participating in the market, can produce economic behaviors or change the economic structure. Instead of fighting alone, they should rely on the power of the network to actively form a relationship network to play a role.

This paper selected nearly all TV dramas from TV stations and three major video websites (iQiyi, YouKu, and Tencent Video) in 2020, using the combination of qualitative and quantitative methods to find the new trend of competition and cooperation between production companies in the TV-drama industry. The research sample selected 487 TV dramas (first broadcast and rebroadcast) played on China's TV channel in 2020, as well as the top 200 Internet dramas (not broadcasted on TV station) on the three major video websites. The list of all production companies was obtained through Baidu Encyclopedia and pull film confirmation, including 492 TV-drama production companies, 293 Internet drama production companies, and 110 companies involved in both TV-drama production and Internet drama production.

### 4.1. Creative Resources and Value Derivative Channels Are Involved in the Competition and Cooperation Relationship by Social Networks

First, content creativity is the foundation of development for TV-drama industry [36]. Only good creativity can generate artistic value. Therefore, starting from the origin of TV-drama production, the relational network begins to exist in the creation stage, and imagination is also outlined in communication with others [37]. Similarly, in the production stage, the relational network, as a strong tacit knowledge, acts on the communication, interaction, and connection of creative production. The city is the creative base of the relational network, and the diversified interpersonal communication and enterprise cooperation foster the development of the TV-drama industry. For this reason, the TV-drama industry in China is mostly gathered in the city to share resources and relationships [38].

In the information age, the connection and network relationship promote the generation of ideas and value realization [39]. Especially, driven by commercial value, cultural and creative industries such as TV dramas are collecting high-quality ideas and resources scattered in society and promoting the positive development of the industry. The “Creative Economy” report released by the Development Research Center of The State Council redefines the Internet plus cultural and creative model, showing the relational network among enterprises, users, and creative people in the creative industry [40]. Many TV-drama production companies focus on online literature platforms in the script-seeking stage, thus discovering creative sources and tapping consumer groups, resulting in the situation that many TV dramas are popular before they are shot.

Secondly, consumers initially focus on goods because of their utility and value. For example, a certain drama is popular mostly because its content elements, plot, actors, or special effects, provide utility and value to the audience, so that the audience is willing to pay time and attention to obtain “value” or “utility.” Utility theory also explains that consumers have a preference sequence for any goods [41], how to order goods? It is based on the relationality of social construction. So, relationships, societies, and values are connected by people's choices.

Almost every TV drama needs promotion to help it succeed nowadays. However, the essence of publicity and promotion is the generalization of the social relational network. For example, many viewers like to watch Dou ban ratings when watching TV dramas, to judge their self-consumption behaviors. This is the obvious guide of the social relational network to mass consumption. Such as video websites, TV-drama “hot value” directly affects advertisers. Therefore, guanxi not only affects the viewing demand of the group, but also affects the marketing activities of the enterprise.

Therefore, the relational network becomes the paradigm of value derivative of TV-drama production companies. The utility and value of TV dramas are no longer limited to the works themselves, but involved in social relations such as media organizations, social platforms, and marketing channels and gathered energy and released energy in the relational network.

### 4.2. The Switch-Based Cooperative Relationship Model Is Constructed in the Competition and Cooperation Adaptation of Enterprises of Social Network

Nowadays, the TV-drama industry is booming, with an annual output of more than 20,000 episodes in China [42]. But only a few can be received and broadcast on the platform. Any TV-drama producing company hopes their production to be broadcast. Therefore, in terms of the common realization of organizational goals, the relational network formed between companies becomes a relational organization that has different market behavior and hierarchical structure. Cultural products such as TV dramas are characterized by a high uncertainty in production and trading process, complex price and pricing indexes, sensitive observation of consumers' consumption, and timely access to market information. Such changeable products are exactly in line with the convenient and complex production response of the relationship network.

In fact, before the Internet era, “project network” based on “project responsibility system” cooperation has been widespread in the field of TV-drama production. Alen carried out research on the agglomeration area of The French Film Industry early on and found that the agglomeration trend of the French film industry was enhanced because employees were frequently redistributed, resources were also migrated on a small scale, film production and production functions were decomposed, and the relationship between enterprises and individuals also built up its network due to production [43].

Li further focused on the cooperation of “Guanxi Circle” among producers, directors, and actors and found that the main body of film production began to show the core dependence on centralization [44]. Nowadays, in the TV-drama production, the cooperation between enterprises is in the mode of crowdsourcing, or the group cooperation network centered on a core enterprise. Each production company plays a role in a different collaborative system, serving different projects, like a “switchboard” that inputs and outputs simultaneously. However, to become a member of any collaborative network, you need to participate in peer competition to gain the opportunity to stabilize the relationship in cooperation.

Through the analysis of samples, 56% (274) TV dramas and 75% (149) Internet dramas are made by two or more joint production. The joint production of TV-drama has become the new normal pattern in the market. Producing companies living in different groups have become a popular investment strategy in the high uncertainty TV-drama investment field. It is also a strategy with a relatively superior earnings ratio. Coproduction is not only a way to reduce investment risk, but also a way to expand your network. In the preparatory period, production stage, distribution and publicity of TV dramas, bundling with strong resources and high-quality projects, not only is the guarantee of broadcast, but also is for maximizing profits.

Among nearly 800 companies with coproduction experience, companies with resources and platform advantages such as China central television (CCTV), Midday Sunshine, Tencent, IQiyi, and YouKu are far ahead in the number of dramas produced (see Table 1). There are also quite a few long-tail companies involved in the production of only one TV series that can be broadcast in 2020. The Matthew effect is obvious in the TV-drama production field, and the competition between small companies will become more brutal.

### 4.3. Resources and Platform Advantages Are the Basis for Enterprises to Demonstrate Their Competitive and Cooperative Capabilities in Social Networks

In the relational network formed based on the production system, the degree of extensive cooperation between production companies is not enough. In the social network study, the overall network density index can reflect the close relationship between network members [45]. Its value is between 0 and 1. The higher the density value is, the closer the relationship between members will be, which also means that the relationship structure can affect the attitude and behavior of members more. For example, if the actual number of nodes in the social network is *n* and the number of connections is *m*, the formula for calculating the overall network density is

(1) $$\begin{array}{c} D=\frac{m}{n\left(n-1\right)}\text{.} \end{array}$$

By calculating, the overall network density of TV-drama production companies is 0.0083 and that of the Internet drama production companies is 0.0116. Therefore, from the perspective of numerical value, the cooperative relationship network between production companies is relatively distant, and there are not many companies that can cooperate.

Therefore, in the TV-drama production market, core enterprises with resources and platforms have extremely strong network centrality and significant market concentration. The total amount and scale of TV dramas produced by leading companies are the largest, and the market is extremely concentrated. For example, the degree centrality value of CCTV in the “TV-Drama” network is as high as 200, and it is the most important enterprise in the whole “TV-Drama” social network. In “Internet Drama,” Tencent and IQiyi ranked the top two among network producers with 67 and 66 degrees of centrality, respectively.

As can be seen from the 2-mode relationship diagram of the top 10 enterprises ranked by the centrality of TV-drama social networks (Figure 2), CCTV is the enterprise with the highest concentration of outbound (red dot) and inbound (blue dot) degrees. Similarly, the 2-mode relationship diagram of Internet drama centrality also shows the same conclusion, with Tencent and IQiyi having the most relationship resources (Figure 3).

### 4.4. Key Position Occupying or Connecting Is the Core of Competitive and Cooperative Relationship of Enterprises in Social Networks

The social network is a complex network based on relationships, which emphasizes multilateral, three-dimensional, and hypergeographic [46]. At present, the strength of internal resources can hardly meet the needs of enterprises to participate in market competition, and enterprises need to establish strong and mutual trust cooperation with the outside more widely than ever before and can maintain long-term stability. Therefore, enterprises urgently need to build external environment and resource utilization channels based on social networks and establish a corporate relationship community that can quickly adapt to market changes and reduce risks through such social networks and break through unilateral cooperation [47].

Resources such as capital, manpower, and information flow extremely fast in the network age. It is not enough for enterprises to rely on each other. They need to participate in the construction of social networks and become nodes or even centers in the network [48]. The “structural hole theory” proposed by Professor Burt [49] further deepens the “weak relation theory” proposed by Granovetter. He points out that the key to the relational network is not how weak the relation is, but how many structural holes are contained in the relation. Hole structure refers to the nonredundant relation between two action subjects or, say more directly, is to make the relational intermediary between two independent networks. It can generate interests and control information; especially in the market competition, the human capital and financial capital are extremely sufficient, and the social capital will become the key to determining success or failure factors. The position of enterprises in social networks is extremely important, which directly determines the acquisition of information and resources and power distribution.

Therefore, starting from Burt's theory of structural holes, if an enterprise wants to maintain a dominant position in the industry, it needs to establish extensive connections and try to become an intermediary in the structural holes to obtain more resources and expand its boundaries. Ding et al. [50] conducted a study on the cooperative network relationship between film production companies. According to the cooperation for production and distribution stages, they found that companies at the core node position could easily obtain resources from other companies and had core advantages in distribution. Although most enterprises are independent subjects of society, they must seek to expand social networks to seize the market for various purposes. Based on the above reasons, the cooperation between TV-drama companies is extremely extensive.

Through the measurement of the “Structure Hole Index” of the sample companies, it is found that, in the relational network of TV-drama production companies, the effective size of CCTV reaches 158.923 (see Table 2), indicating that it has the largest influence in the whole network. Tencent (effective size: 59.681) and IQiyi (effective size: 56.139) (see Table 3) are also the most influential companies in the relationship network. Effective size is an index to measure the influence of nodes, and the calculation formula is as follows:

(2) $$\begin{array}{c} {ES}_{I}=\underset{j}{\sum }\left(1-\underset{q}{\sum }P_{iq}P_{jq}\right)=n-\frac{1}{n}\underset{j}{\sum }\underset{q}{\sum }P_{jq}\text{,} \end{array}$$

*n* represents the degree of node *i*, *j* represents the adjacent node of node *i*, and *q* represents the common adjacent node of node *i* and node *j*. *P*_*iq*_ and *P*_*jq*_ represent the weight proportion of node *q* in the adjacent nodes of node *i* and node *j*, respectively.

Similarly, the index of constraint indicates the closeness between nodes. The lower the index is, the more open the network is, and the more the number of master structure holes is. In the network of TV-drama production, there are 20 companies whose constraint is less than 0.15, indicating that these 20 companies hold most of the structural holes in the network. Among them, 5 companies whose constraint is less than 0.1 are key opinion leaders in the relational structure. However, in the relational network of Internet drama production companies, only three companies have a constraint less than 0.15, which are the three major video website platforms. The scale and resources of these three companies are in an absolute leading position in the relationship in Internet drama production and control the social capital in the network.

### 4.5. The Reconstruction of Cooperation Mechanism in Clique Structure Is the Key to Establishing a Competitive Cooperation Relationship

Whether to establish a social network relationship or maintain the original connected cooperative relationship has always been a topic of constant discussion in the process of establishing a cooperation mechanism. Many entrepreneurs and academics also think that it is safer to keep the old relationship. Because, on the one hand, the original relationship is also a resource acquisition channel, and it works well, there is no need to destroy it; on the other hand, partners in the original relationship and cooperation have experience in terms of ability, stability, and value convergence, which reduces the risk of cooperation. But in a highly competitive market, especially in TV industry with so many unaired episodes produced each year, maintaining the original relationship can lose a lot of market opportunities.

Gulati et al. [51] divided enterprises into three types of ways to enter social networks: structure embedding, location embedding, and relationship embedding. Structure embeddings indicate that enterprises play a mediating role. Location embedding determines the convenience of obtaining information; relationship embedding represents the possibility of cooperation between enterprises. Therefore, the enterprise cooperation mechanism in social networks is no longer a simple connection, but a search for location, relationship, and structure. In the TV-drama industry, the core production company occupies the central position in the relational network and forms a certain network clique. For example, when a TV station participates in the production of a TV series, many TV companies want to cooperate with it because it can ensure the broadcast of the series. The position of the TV station in the social network will be in the central position, especially the strong TV station. Through empirical analysis, based on the extended application of the concept of minimal group in the social network theory, 320 cliques have been formed in the relational network between the overall TV-drama production companies, among which there are as many as 112 cliques with CCTV as the core member, and 20 cliques with Tencent as the core. In the overall network of Internet drama production companies, 88 cliques have formed, among which 20 are centered on Tencent and IQiyi, and 15 are centered on Youku. In the clique, the core enterprise has an extremely high intermediary ability and has strong market control in terms of resources, technology, capital, talent, communication, and other aspects and can even directly determine whether the drama can be broadcast.

In social network analysis, the centrality of mediation is often used to describe the mediating capability of nodes, which reflects the role of a node as a bridge between other nodes in the network. The higher the degree, the greater the resource control and intermediary value. In TV-drama social network, CCTV (mediation centrality: 42.837) is the highest mediating capability (see Table 4). And in Internet drama social network, Tencent, iQiyi, and Youku are similarly influential (see Table 5). From the data analysis, it can be clearly recognized that the key to the success of small- and medium-sized companies is to participate in the clique of high mediation companies and reshape the cooperation mechanism with clique standards, especially in the clique occupied by the head enterprise, and the exchange of knowledge and information between companies can also become an important weight for enterprises to participate in the competition. It can be seen from the latest IPO of film and television enterprises declaration that the relationship capital with high intermediary core enterprises has become the dominant feature in the declaration.

### 4.6. Seeking the Best Position in the Social Network and Trying to Find Heterogeneous Partners

In the TV-drama market, there are many homogeneous companies, so there will be many competitors for the same job, which may lead to the failure of cooperation due to fierce competition, and even the hidden danger of being replaced during the cooperation. So, what can be done to mitigate the conflict of being replaced in social network partnerships? From the perspective of relationship, the company can try to explore the processing of network location and relationship.

First of all, the previous study found that, in the TV-drama production cooperation network, the overall and partial network characteristics as well as the position of the enterprise in the social network will affect the advantages of the enterprise in different competitive environments. Therefore, enterprises need to find a better position in the cooperation network to enhance their competitiveness. Through the improvement of the company's strength, capital, resources, reputation, and other factors, the company will have more advantages to choose perfect partners and even become the main body with structural holes in the social network, so as to gain stronger competitiveness.

Secondly, enterprises should be able to participate in social network cooperation and, at the same time, be able to judge the market atmosphere. Both social circles need to be actively involved, so that enterprises can choose partner freely in the TV-drama market. Although the location advantage brought by the cooperative relationship network can enhance the competitive strength of enterprises, the income of TV-drama project is not entirely determined by the social network. It also needs to refer to the market environment, such as market entry barriers, popularity of TV-drama content type, audience demand, and other factors.

Finally, most conflicts in social networks are caused by competition. Therefore, on the one hand, enterprises not only need to enhance their competitiveness, but also need to seek for heterogeneous enterprises to cooperate, having a unique role in the cooperative relationship network. Because the nonequivalence relationship of structure means that resources and information are complementary between companies, cooperation will not reduce their respective competitive advantages and can better play the overall team cooperation effect and reduce contradictions.

## 5. Conclusion and Reflection

In the process of production, communication, and consumption, many unknown variables may affect the meaning of social production, such as potential relationship. Therefore, social networks may provide a new cognitive perspective on the production process reengineering, business model innovation, organizational form change, and national policy change in the cultural industry.

### 5.1. Subject Cognition Reconfirmation: Transform from Subject Connection to Subject Relation Construction

From the perspective of a relational network, the connection of TV-drama industry can be regarded as the most extensive connection. The development of TV-drama industry not only depends on the expansion of enterprises themselves, but also needs to build a relational network with the central company as the core operation. Judging from the relational structure between “TV-drama” and “Internet drama,” there are not many core companies that can build a network of relationships. Although there are a large number of companies in industries, the company that has resources, capital, and platform is one of the few, like CCTV, Hunan TV, Midday Sunshine, Tencent, and so on. These big institutions or companies are extremely popular because most companies are willing to work with them. Instead of cooperation between small companies being very little, the universality of relations in the network cooperation relationship is not prominent. Therefore, the key for the participants is to walk into the construction of the subject relationship and find the best position to obtain more resources and capital. Of course, the choice of path in relation to exploration is important, not the initiative to implement relational structures and also the need to gradually accumulate in the development, especially to find the key subject of product characteristics, such as CCTV on policy, thoughts lead, content creation, and more preference; if you want to establish relations with CCTV, on the setting characteristics, direction can be known diligently.

### 5.2. Reexploration of Path Cognition: Transformation from Linear Thinking to Relational Thinking

There are direct or indirect relations between various subjects in the clique, and the cooperation will be relatively close, and even a closed cycle of multiple cooperation will appear. And with many small companies in the partnership, some only cooperate once, and some never cooperate, resulting in the fierce TV-drama market being marginalized, or even difficult to survive.

Therefore, for better digging resources and seeking innovation in TV-drama social network, it needs industry practitioners to change original linear cooperation thinking into a system of thinking, not only considering the competition, but also considering how to cooperate. Because cooperation could make the segmentation unit in the network structure show new properties and new features, to realize the efficient allocation of resources, this kind of cooperation is not only to break through the inherent connection between clique members, but also to plan the overall network relationship structure with systematic thinking and to establish a wide cooperative relationship with the company with high centrality as the intermediary, so as to produce rich and valuable TV dramas for the society.

### 5.3. Redeconstruction of Power Cognition: Transformation from Absolute Center to Decentralized Center

Enterprises with strong resource advantages occupy the key position in the market and have the absolute power of discourse in the industry. But in the network, the production of any product will not be affected by contract power. They will rely on the production capacity of the network nodes, the ability to change the relationship, or the ability to organize network. In the future network, the monopoly body will disappear and be replaced by the main body of different importance whose connectivity is more important than the production capacity.

In the network production rule, the node which can connect, and the production will be distributed in every link of TV-drama industry ecology. For example, these platform companies, Tencent and TouTiao, will make the rules in their own subgroup, extending outward at the same time, to connect more and more central nodes to improve the competitive ability of the group. In the future, the companies will be able to obtain more data, information, capital, human resources, and other diversified capabilities if they are able to obtain a location in the decentralized center layout. Moreover, enterprises should clearly realize that the power center is fluid, and the advantages of the platform may gradually disappear. In order to control the relationship network for a longer time, central enterprises need to constantly set themselves at the center of the relationship structure, which also poses challenges to the strength of enterprises.

With whom, how to connect, and how they are structured are all factors that affect the relocation of economic activity. The interaction between producers, consumers, and channel merchants is more frequent, and the connection is from series to parallel, so absolute control is deprived. Any individual in the relationship may change the relationship structure and generate huge energy. For example, online communities activate individual productivity, sharing economy activates the utilization of idle resources, and timeliness and mobility become the existence of network relations. Competition and cooperation in the TV-drama industry will get rid of the absolute center and establish the relative center, and the dominant ability of TV stations and video platforms will be further reduced. The traditional media are no longer the master of TV play terminal, and the video websites have begun to move from competition to cooperation. The mechanism of these phenomena is related to the mature development of the relational network. The situation of TV-drama industry is relatively complicated, and more diversified, decentralized centers will be formed in the future, such as content center, capital center, talent center, and production center. Both individuals and organizations need to place themselves in a large, interactive, and interconnected relationship network. This also provides a broad direction for follow-up studies to consider the role of social network relationships more widely from different roles in the production chain such as content, capital, and human resources.

## Figures and Tables

**Figure 1:** Relationship model of information delivery and sharing in the TV-drama industry supply chain.

**Figure 2:** Relationship of top 10 centrality companies in the TV-drama social network.

**Figure 3:** Relationship of top 10 centrality companies in the internet drama social network.

**Table 1:** List of the top 10 producers in terms of number of coproductions in 2020.

NO.	TV drama		Internet drama	
	Producing number (unit)	Producer	Producing number (unit)	Producer
1	136	CCTV	39	TENCENT
2	13	HUACE FILM	39	IQIQI
3	13	PERFECT MOVIE	34	YOUKU
4	12	TENCENT	10	HAPPY SUNSHINE
5	11	MIDDAY SUNSHINE	7	HUACE FILM
6	10	OMNIJOI MEDIA	6	NEW MEDIA CHENGPIN
7	10	SMG PICTURES	5	WANDA MOVIE
8	9	YOUKU	5	PERFECT MOVIE
9	9	SHANDONG FILM	5	ALIBABA FILM
10	8	HIBN	4	STRAW BEAR

**Table 2:** Key companies in the structure hole of TV-drama production company.

No.	Name	Effective size	Constraint
1	CCTV	158.923	0.016
2	IQIYI	34.556	0.069
3	TENCENT	33.072	0.063
4	OMNIJOI MEDIA	25.192	0.082
5	H&R CENTURY	19.158	0.098
6	MANGO STUDIO	18.231	0.111
7	SMG PICTURES	18.079	0.109
8	NANJING TV	17.190	0.106
9	HUACE FILM	13.409	0.115
10	WANDA MOVIE	13.288	0.117

**Table 3:** Key companies in the structure hole of internet-drama production company.

No.	Name	Effective size	Constraint
1	TENCENT	59.681	0.033
2	IQIYI	56.139	0.039
3	YOUKU	39.448	0.052
4	PERFECT MOVIE	11.538	0.166
5	NEW MEDIA CHENGPIN	10.463	0.184
6	WANDA MOVIE	8.548	0.194
7	HUAYI BROTHERS	7.088	0.233
8	GOLDEN SHIELD TV CENTER	7.000	0.215
9	ZHONGHUI MOVIE	7.000	0.251
10	HAPPY SUNSHINE	6.714	0.177

**Table 4:** Centrality of mediation of subgroup key companies in TV-drama social network.

No.	Name	Subgroup centrality of mediation
1	CCTV	42.837
2	TENCENT	5.775
3	IQIYI	4.806
4	YOUKU	4.448
5	OMNIJOI MEDIA	4.290
6	PERFECT WORLD	4.249
7	H&R CENTURY	4.231
8	SHANDONG TV	3.920
9	PHOENIX LEGEND	3.462
10	SMG PICTURES	2.692

**Table 5:** Centrality of mediation of subgroup key companies in internet drama social network.

No.	Name	Subgroup centralityof mediation
1	TENCENT	19.520
2	IQIYI	16.828
3	YOUKU	13.277
4	WANDA MOVIE	4.889
5	PERFECT MOVIE	4.131
6	GOLDEN SHIELD TV CENTER	3.968
7	HUAYI BROTHERS	3.507
8	TIAN HAO	2.970
9	NEW MEDIA CHENGPIN	2.698
10	MANGO TV	2.169

## Data Availability

The data that support the findings of this study can be obtained from the corresponding author upon reasonable request.

## References

[1] Chen L. Q. (2016). Research on we-media people in the era of social media. *Frontiers*.

[2] Fei X. T. (2008). *Rural China*.

[3] Zhang F. H. (2010). Conceptual model and empirical analysis of the impact of network embedding on enterprise innovation performance [J]. *China Industrial Economics*.

[4] Castells M., Fernandez-Ardevol M., Qiu J. L., Sey A. (2009). *Mobile Communication and Society: A Global Perspective*.

[5] He J. L., Huang X. J., Si Y. F. (2018). Local embedment of industrial clusters and global production network link: a case study of Shanghai Cultural and creative industry Park [J]. *Geographical Research*.

[6] Xin X. R., Zeng G. (2019). Research on Chinese film production industry based on network structure [J]. *Economic Geography*.

[7] Wen C., Zhang Q. Q., Su X. (2019). Research on the city network based on the Division of labor of Value chain of Chinese film industry. *Human Geography*.

[8] Lu H. Y. (2016). *Study on the Network Structure of China’s TV Industry and its Impact on the Development of Regional Industries [D]*.

[9] Johns J. (2010). Manchester’s film and television industry: project ecologies and network hierarchies. *Urban Studies*.

[10] Bar L. (2020). From corporate aggregation to relational network: re-understanding the creative industry in the Internet age. https://lujuba.cc/en/289700.html.

[11] Bucklin L. P., Sengupta S. (1993). Organizing successful Co-marketing alliances. *Journal of Marketing*.

[12] Lu W. M., Kweh Q. L., He D. S., Shih J. M. (2017). Performance analysis of the cultural and creative industry: a network‐based approach. *Naval Research Logistics*.

[13] Turok I. (2003). Cities, clusters and creative industries: the case of film and television in Scotland. *European Planning Studies*.

[14] Wasserman S., Faust K. (1994). *Social Network Analysis: Methods and Applications*.

[15] Barabási A.-L., Jeong H., Néda Z., Ravasz E., Schubert A., Vicsek T. (2002). Evolution of the social network of scientific collaborations. *Physica A: Statistical Mechanics and Its Applications*.

[16] Cross R., Parker A., Prusak L., Borgatti S. P. (2001). Knowing what we know. *Organizational Dynamics*.

[17] Cross R., Borgatti S., Parker A., Cross R., Parker A., Sasson L. (2003). Making invisible work visible. *Networks in the Knowledge Economy*.

[18] Kim Y., Choi T. Y., Yan T., Dooley K. (2011). Structural investigation of supply networks: a social network analysis approach. *Journal of Operations Management*.

[19] Park S. B., Oh K. J., Jo G. S. (2011). Social network analysis in a movie using character-net. *Multimedia Tools and Applications*.

[20] Rosenquist J. N. (2011). Lessons from social network analyses for behavioral medicine. *Current Opinion in Psychiatry*.

[21] Baah C., Opoku Agyeman D., Acquah I. S. K. (2021). Effect of information sharing in supply chains: understanding the roles of supply chain visibility, agility, collaboration on supply chain performance. *Benchmarking: An International Journal*.

[22] Mageto J. (2021). Big data analytics in sustainable supply chain management: a focus on manufacturing supply chains. *Sustainability*.

[23] Jelti F., Allouhi A., Büker M. S., Saadani R., Jamil A. (2021). Renewable power generation: a supply chain perspective. *Sustainability*.

[24] Wiengarten F., Humphreys P., Cao G., Fynes B., McKittrick A. (2010). Collaborative supply chain practices and performance: exploring the key role of information quality. *Supply Chain Management: International Journal*.

[25] Lee H. L., So K. C., Tang C. S. (2000). The value of information sharing in a two-level supply chain. *Management Science*.

[26] Kulp S. C., Lee H. L., Ofek E. (2004). Manufacturer benefits from information integration with retail customers. *Management Science*.

[27] Yu H., Zhen X. P. (2012). Two-stage online distribution strategy of emergency material. *Systems Engineering-Theory & Practice*.

[28] Bourland K. E., Powell S. G., Pyke D. F. (1996). Exploiting timely demand information to reduce inventories. *European Journal of Operational Research*.

[29] Chen F., Drezner Z., Ryan J. K., Simchi-Levi D. (2000). Quantifying the bullwhip effect in a simple supply chain: the impact of forecasting, lead times, and information. *Management Science*.

[30] Paik Y., Kim Y., Rawley E. (2018). Vertical Collaboration and the Performance of Knowledge-Based Products: Evidence from the Korean TV Drama Industry.

[31] Lowry P. B., Zhang D., Zhou L., Fu X. (2010). Effects of culture, social presence, and group composition on trust in technology‐supported decision‐making groups. *Information Systems Journal*.

[32] Nestle V., Täube F. A., Heidenreich S., Bogers M. (2019). Establishing open innovation culture in cluster initiatives: the role of trust and information asymmetry. *Technological Forecasting and Social Change*.

[33] Lipyanina H., Sachenko A., Lendyuk T., Nadvynychny S., Grodskyi S. (2020, April). Decision tree based targeting model of customer interaction with business page. *CMIS*.

[34] Scherer F. M. (2007). *How Conservative Economics Has Influenced Antitrust*.

[35] Werron T. (2014). On public forms of competition. *Cultural Studies ↔ Critical Methodologies*.

[36] Zhu Y., Keane M., Bai R. (2008). *TV Drama in China*.

[37] Gummesson E. (1998). Productivity, quality and relationship marketing in service operations. *Hand Buch Dienstleistungs Management*.

[38] Huang A. L. (2012). *A Study of Beijing’s Competitive Advantage as an Emergent media Capital (Doctoral Dissertation)*.

[39] Agustina Y., Winarno A., Pratikto H., Narmaditya B. S., Filianti F. (2020). A creative economy development strategy: the case of Trenggalek creative network for Trenggalek Regency, Indonesia. *The Journal of Asian Finance, Economics and Business*.

[40] China Economic Culture Industry China puts forward the concept of “creative economy” for the first time, a new era of cultural and creative industry?. https://www.sohu.com/a/131064987_488901.

[41] Nocella G., Boecker A., Hubbard L., Scarpa R. (2012). Eliciting consumer preferences for certified animal‐friendly foods: can elements of the theory of planned behavior improve choice experiment analysis?. *Psychology and Marketing*.

[42] Zhu Y. (2013). *Television in post-reform China: Serial Dramas, Confucian Leadership and the Global Television Market*.

[43] Allen R. C. (2010). Getting to going to the show. *New Review of Film and Television Studies*.

[44] Li B., Chen L. Y. (2015). From professional logic to capital logic: a social network analysis of the main body of Chinese film production: based on the cooperation relationship between filmmakers and directors from 2004 to 2014. *International press*.

[45] Horan W. P., Subotnik K. L., Snyder K. S., Nuechterlein K. H. (2006). Do recent-onset schizophrenia patients experience a “social network crisis”. *Psychiatry: Interpersonal and Biological Processes*.

[46] Li G., Hu J., Song Y., Yang Y., Li H. J. (2019). Analysis of the terrorist organization alliance network based on complex network theory. *IEEE Access*.

[47] Sturgeon T. J. (2002). Modular production networks: a new American model of industrial organization. *Industrial and Corporate Change*.

[48] Borgatti S. P., Li X. (2009). On social network analysis in a supply chain context. *Journal of Supply Chain Management*.

[49] Burt R. S. (1992). *The Social Structure of competition*.

[50] Ding H. Q., Wu Y. W. (2018). Research on cooperation network of Domestic film Production and distribution. *News Front*.

[51] Gulati R. (1999). Network location and learning: the influence of network resources and firm capabilities on alliance formation. *Strategic Management Journal*.

